The article "Application of Mathematical Modeling in Cost Control of Medical Equipment Procurement in Public Hospitals" was retracted in 2023. Reasons: unreliable results or conclusions; concerns about the data; concerns about the results or conclusions; concerns about the peer review.

# Application of Mathematical Modeling in Cost Control of Medical Equipment Procurement in Public Hospitals

**DOI:** 10.1155/2022/3425873

**Published:** 2022-07-07

**Authors:** Lihong Chen

**Affiliations:** Department of Procurement Center, Shanghai Tenth People's Hospital, Shanghai 200072, China

## Abstract

The purpose of this study is to strengthen the procurement management of public hospitals and ensure the quality of medical equipment. In this paper, combined with the procurement process of medical equipment in public hospitals, on the basis of RFID technology, a JRP model of random demand for medical equipment procurement in public hospitals is established. At the same time, according to the type and quantity of decision variables, the DE solution algorithm is redesigned, and based on the support of the algorithm, a mathematical model for cost control of medical equipment procurement in public hospitals is established. It can be seen from the analysis results that the cost control system for medical equipment procurement in public hospitals based on the mathematical model proposed in this paper can play an important role in public hospital equipment procurement and promote the standardized operation of public hospital procurement management.

## 1. Introduction

Medical equipment investment is an important part of hospital construction planning. As the hospital now advocates the business model of “supporting doctors with skills,” the increase in various surgeries and inspection items will inevitably increase the investment in related medical equipment. How to effectively control the cost of medical equipment procurement, that is, how to balance the expenditure and recovery of funds in this area, has become a common concern. This paper discusses how to effectively control the procurement cost of medical equipment in a second-class A-level hospital, dynamically observes various constituent factors of the procurement cost of medical equipment, and puts forward many insights and methods to effectively control the procurement cost of medical equipment. Moreover, the effectiveness of the specific content of the comprehensive equipment procurement system to reduce the procurement cost is discussed. The results show that adopting appropriate bidding procurement methods and establishing a perfect and standardized procurement system are most conducive to scientifically controlling equipment procurement costs, thereby reducing the overall cost of hospitals. Therefore, controlling the procurement cost of medical equipment and making it continue to decrease is one of the important and direct means to reduce the total cost of the hospital and increase the profit.

The article "Application of Mathematical Modeling in Cost Control of Medical Equipment Procurement in Public Hospitals" was retracted in 2023. Reasons: unreliable results or conclusions; concerns about the data; concerns about the results or conclusions; concerns about the peer review.

Budget management is the main method for the hospital to implement the refined management of large medical equipment. It is to control the activities of various kinds of medical equipment in the hospital and to demonstrate, purchase, manage, and coordinate the various resources of the hospital. Budgeting is also a comprehensive management model, which requires hospitals to forecast and arrange future hospital equipment procurement and distribution in light of business requirements and development, comprehensively consider the hospital's capital status and financial resources, demonstrate and analyze medical equipment, and make overall planning for equipment budgets. By strengthening budget management, it can provide support for the follow-up equipment management work. When carrying out equipment management, hospitals should carry out equipment management according to the requirements of budget management, strengthen equipment procurement, maintenance, tracking, investigation, assessment, etc., to realize the overall arrangement of budget management, and combine with budget performance assessment to ensure the smooth completion of equipment management goals. The economic benefit analysis of large-scale medical equipment is the foundation of equipment budget management, and it is also the basis for equipment budget decision-making and review. By strengthening the application and benefit investigation and analysis of large-scale medical equipment, it can provide data reference for the deployment and management of hospital equipment and ensure the quality of equipment management.

According to the procurement process of public hospital medical equipment, this paper establishes a mathematical model of public hospital medical equipment procurement and controls the procurement cost of public hospital medical equipment through the intelligent model.

## 2. Related Work

No enterprise can operate independently from procurement activities. According to Porter's value chain profits, as long as the business remains in operation, then the purchasing activity is bound to happen. That is to say, enterprises must pay suppliers a certain amount of funds in exchange for goods and services, that is, to meet and maintain the operation of the organization through procurement activities [1]. In simple terms, procurement is the necessary economic activity for an enterprise to obtain the materials it needs, including a series of operations such as planning, decision-making, purchasing, tracking, acceptance, transportation, and storage [2]. Therefore, in a narrow sense, procurement is the purchase behavior of products or services according to their own needs for the purpose of operation and production [3]. From a broad perspective, procurement is an economic activity in which an enterprise obtains ownership of resources through multiple channels and methods, cyclically and continuously, and its purpose is to meet all of its own needs. With the blowout reform of science and technology and the in-depth development of regional economic integration, all enterprises today are faced with extremely fierce market competition and changing consumer market. Enterprises need to further shorten the reaction time to the market and continuously improve the quality of their own products, but also simultaneously reduce production and operation costs, so as to maintain a good capital flow and ensure the survival and competitiveness of enterprises [4]. Procurement activities are one of the important links in the operation of enterprises, and procurement costs account for about 60% of operating costs. If the procurement cost can be effectively controlled, it can directly reduce the operating cost of the enterprise and indirectly create value for the enterprise. Therefore, how to control procurement costs has become an extremely important factor for the survival and competitiveness of today's global enterprises [5].

The article "Application of Mathematical Modeling in Cost Control of Medical Equipment Procurement in Public Hospitals" was retracted in 2023. Reasons: unreliable results or conclusions; concerns about the data; concerns about the results or conclusions; concerns about the peer review.

With the continuous updating of procurement management theory, more and more enterprises use it for literature in the practice of procurement activities and gradually upgrade their procurement from traditional mode to strategic procurement. The core of transformation and upgrading is to comprehensively summarize and analyze the cost of product purchase, use, quality inspection, and maintenance in procurement activities through strategic procurement management and further strengthen cost control [6]. Literature [7] established a TCO model and analyzed the important material procurement activities of many companies through empirical research methods. Finally, by using the TCO model, it is confirmed that TCO can help enterprises select suitable suppliers, optimize supplier management, and strengthen cost management. The author further suggests that the TCO model can be promoted to leading enterprises in various industries, which will help these leading enterprises maintain their core competitiveness. Literature [8] proposed that TCO (full name total cost of ownership) is a concept of total cost integration. In the application of this theory in corporate procurement activities, it refers to all costs in the procurement process, including but not limited to ordering, acceptance, use, maintenance, and defect disposal. TCO can be used as a procurement tool for enterprises to better analyze all the costs incurred between enterprises and suppliers when the procurement relationship occurs. From the perspective of the time dimension of the procurement activities, the prepurchase cost is all the costs before the enterprise purchase order is determined, including the confirmation of procurement requirements, the development and selection of suppliers, and the internal communication between the enterprise demand department and the procurement department [9]. The interim cost of procurement is the relevant cost incurred when confirming the purchase order of the enterprise, including the cost of purchase price, transportation, delivery, tax payment, inspection, tracking, and after-sales. The postprocurement cost is the cost incurred at the end of the procurement activity cycle, including the cost of concession receipt, repair cost, maintenance, and upkeep [10].

The article "Application of Mathematical Modeling in Cost Control of Medical Equipment Procurement in Public Hospitals" was retracted in 2023. Reasons: unreliable results or conclusions; concerns about the data; concerns about the results or conclusions; concerns about the peer review.

Literature [11] starts from the TCO theory and studies multiple supplier selection models, focusing on the distinction between the hierarchical model and the mathematical programming model. At the same time, through the method of empirical research, it demonstrates the practicability of the multi-item model in procurement activities. The author stated in the article that the mathematical programming model is more suitable for the management of suppliers' selection in procurement activities, and this multi-item model can help companies obtain more accurate procurement costs. Literature [12] empirically analyzes the company's own procurement strategy and overall procurement cost based on historical procurement cost data and suppliers' procurement performance. The author uses a mathematical programming model to help companies select suitable suppliers and further reduce their overall procurement costs. Literature [13] studies the shortcomings of ABC in selecting and evaluating suppliers. The authors restate the total supplier cost of the procurement process in the article, including the purchase price of the goods, the associated normal operating costs, and additional operating costs due to product defects. On this basis, empirical analysis is carried out through mathematical models, which improves the scientificity and objectivity of supplier selection and evaluation. Literature [14] takes the three dimensions of suppliers, enterprise purchase orders, and purchased products as the research objects and studies the selection cost of suppliers through quantitative analysis. The author makes full use of the TCO theory to construct a data model for cost structure analysis and uses a scientific method to solve the problem of supplier selection and purchase order allocation. Literature [15] quantifies the hidden procurement cost and establishes a comprehensive evaluation index system for the problem of more accurate selection of the best supplier. In this quantitative model, procurement-related factors such as procurement quality, procurement time, and delivery punctuality are fully considered, and the total procurement cost is calculated to improve the accuracy of supplier selection. Literature [16] believes that the best way to evaluate, analyze, and select suppliers is to use the TCO model. In the procurement practice of the enterprise, the TCO model can help the enterprise to better reduce the overall procurement cost, directly improve the profitability of the enterprise, and then ensure the comprehensive competitiveness of the enterprise from the perspective of operating benefits.

The article "Application of Mathematical Modeling in Cost Control of Medical Equipment Procurement in Public Hospitals" was retracted in 2023. Reasons: unreliable results or conclusions; concerns about the data; concerns about the results or conclusions; concerns about the peer review.

## 3. Mathematical Modeling of Procurement Cost Control

Under the periodic inspection strategy, the set inventory level is checked regularly, and the ordering process occurs when the inventory level is reduced to a certain level (minimum service level). The goal of inventory levels is to meet customer demand within the inspection cycle T and order lead time. The safety stock ST_*i*_ for different commodities is usually denoted ${\text{ST}}_{i}=z_{i}\sigma_{i}\sqrt{k_{i}T+L}$. Among them, *z*_*i*_ is the service level factor, *σ*_*i*_ is the standard deviation of the demand forecast error of commodity *i*, *k*_*i*_ is the joint procurement frequency of commodity *i*, and *L* is the order lead time. Multiplying the order lead time by the inventory cost of the classic JRP constitutes the inventory cost of the random demand, which is the basic random JRP and the basis for the construction of the random JRP in this paper.

The research on random demand JRP decision based on RFID technology has the following characteristics:

1. Based on the deterministic JRP, it is the first attempt to establish a JRP model based on the random demand of RFID technology. Using the link between RFID technology investment and RFID return on investment, it links the investment of RFID technology in the JRP process and the impact of RFID technology on JRP cost. Moreover, it takes the lowest total cost of JRP for RFID investment as the research goal and improves the procurement efficiency of random JRP and the JIT efficiency in the process of inventory management
2. It reselects the parameters of the DE algorithm and designs the solution process. The DE algorithm is designed according to the type and number of decision variables of random JRP and the structure of the model, and the sensitivity analysis of the parameters of the algorithm is carried out
3. It solves the optimal investment level of RFID technology and improves the efficiency under the optimal investment level and analyzes the impact of its procurement cost and inventory cost, as well as the reasonable investment scale of RFID. Moreover, it examines the impact of parameter changes on RFID technology investment. Similar to the process of determining JRP, the schematic diagram of the JRP model under random demand conditions is shown in Figure 1

The JRP model of stochastic demand is also based on the JRP of deterministic demand, and the stochastic JRP still takes the total cost as the objective function, which is composed of inventory cost and joint procurement cost. The cost of joint procurement of deterministic JRP is the joint procurement cost of stochastic demand JRP model. It sets the warehouse's maximum inventory level and determines the inventory cost and out-of-stock cost of the JRP model of demand based on the distribution of random demand. These two costs are described in three sections below.

1. Joint procurement cost

According to the joint ordering cost of the determined demand, JRP is composed of the main ordering cost *S* and the secondary ordering cost *s*_*i*_; the corresponding random demand JRP annual ordering cost *s*_*i*_ is [17]:

(1) $$\begin{array}{c} C_{o}=\frac{S}{T}+\overset{n}{\underset{i=1}{\sum }}\left(\frac{s_{i}}{k_{i}T}\right)=\frac{1}{T}\left(S+\overset{n}{\underset{i=1}{\sum }}\left(\frac{s_{i}}{k_{i}}\right)\right). \end{array}$$

(2) Inventory cost

Referring to the inventory model of a single commodity, after the order for commodity *i* is placed, after the lead time *L*_*i*_, the warehouse will receive the ordered commodity that has reached the maximum inventory level *R*_*i*_ of commodity *i*. In the mode of joint procurement, if the initial inventory level of commodity *i* is *R*_*i*_ − *D*_*i*_*L*_*i*_, and if the procurement frequency of commodity *i* is *k*_*i*_, the order for this commodity will be issued at time *k*_*i*_*T*, and the order will be received at time *k*_*i*_*T* + *L*_*i*_. Therefore, the inventory level of commodity *i* in the central warehouse before the arrival of the goods is *R*_*i*_ − *D*_*i*_(*k*_*i*_*T* + *L*_*i*_). Therefore, the average inventory level $\bar{Q_{i}}$ of commodity *i* in the central warehouse in time *k*_*i*_*T* + *L*_*i*_ is

(2) $$\begin{array}{c} \bar{Q_{i}}=\frac{1}{2}\left[\left(R_{i}-D_{i}L_{i}\right)+\left(R_{i}-D_{i}\left(k_{i}T+L_{i}\right)\right)\right]=R_{i}-D_{i}\left(\frac{L_{i}+k_{i}T}{2}\right). \end{array}$$

We assume that the demand for all purchased commodities is independent and identically distributed, and random demand follows a Brownian motion process. Moreover, under the premise that the decision variables *k*_*i*_ and *T* are determined, in the demand period of *k*_*i*_*T*, the demand for commodity *i* follows a normal distribution, and its corresponding mean and standard deviation are expressed as *E*(*x*_*i*_, *k*_*i*_*T*) = *D*_*i*_*k*_*i*_*T* and Var(*x*_*i*_, *k*_*i*_*T*) = *δ*_*i*_*k*_*i*_*T*, respectively, and its probability density function is *f*(*x*_*i*_, *k*_*i*_*T* + *L*_*i*_).

The article "Application of Mathematical Modeling in Cost Control of Medical Equipment Procurement in Public Hospitals" was retracted in 2023. Reasons: unreliable results or conclusions; concerns about the data; concerns about the results or conclusions; concerns about the peer review.

Therefore, the maximum inventory level of a commodity is equal to the expected demand plus the amount of safety stock in the safety period. Considering that the lead time of commodity *i* is *L*_*i*_, the maximum inventory level of commodity *i* in each purchasing cycle is expressed as [18]

(3) $$\begin{array}{c} R_{i}=D_{i}\left(k_{i}T+L_{i}\right)+{\text{z}}_{i}\sqrt{\delta_{\text{i}}\left(k_{i}T+L_{i}\right)}. \end{array}$$

Among them, *f*(*z*_*i*_) and *F*(*z*_*i*_) are the probability density function (PDF) and cumulative distribution function CDF of the standard normal distribution corresponding to commodity *i*, respectively. Then, the inventory holding cost *C*_*H*_ is expressed as

(4) $$\begin{array}{c} C_{H}=\overset{n}{\underset{i=1}{\sum }}h_{i}\left[R_{i}-D_{i}\left(\frac{L_{i}+k_{i}T}{2}\right)\right]=\overset{n}{\underset{i=1}{\sum }}h_{i}\left[\frac{1}{2}D_{i}\left(k_{i}T\right)+{\text{z}}_{i}\sqrt{\delta_{\text{i}}\left(k_{i}T+L_{i}\right)}\right]. \end{array}$$

When the demand for commodity *i* is greater than the maximum inventory, the warehouse will be out of stock. In the out-of-stock mode under the regular inspection strategy, it will cause the corresponding out-of-stock cost to the central warehouse. The total out-of-stock cost *C*_*s*_ is expressed as [19]

(5) $$\begin{array}{c} C_{s}=\overset{n}{\underset{i=1}{\sum }}\pi_{i}\int_{R_{i}}^{\infty }\left(x_{i}-R_{i}\right)f\left(x_{i},k_{i}T+L_{i}\right)\frac{{dx}_{i}}{k_{i}T}=\overset{n}{\underset{i=1}{\sum }}\frac{\pi_{i}}{k_{i}T}\sqrt{\delta_{\text{i}}\left(k_{i}T+L_{i}\right)}\int_{{\text{z}}_{i}}^{\infty }\left(y-z_{i}\right)f\left(y\right)dy=\overset{n}{\underset{i=1}{\sum }}\frac{\pi_{i}}{k_{i}T}\sqrt{\delta_{\text{i}}\left(k_{i}T+L_{i}\right)}\left(\int_{{\text{z}}_{i}}^{\infty }yf\left(y\right)dy-\int_{{\text{z}}_{i}}^{\infty }z_{i}f\left(y\right)dy\right)=\overset{n}{\underset{i=1}{\sum }}\frac{\pi_{i}}{k_{i}T}\sqrt{\delta_{\text{i}}\left(k_{i}T+L_{i}\right)}\left(f\left({\text{z}}_{i}\right)-{\text{z}}_{i}\left(1-F\left({\text{z}}_{i}\right)\right)\right). \end{array}$$

(3) Total cost of joint procurement

By constructing purchasing cost, inventory cost, and out-of-stock cost, the stochastic JRP total cost TC with *K*, *T*, and z_*i*_ as decision variables is the sum of the above three costs:

(6) $$\begin{array}{c} \text{TC}\left(K,T,z_{i}\right)=C_{o}+C_{H}+C_{S}=\frac{1}{T}\left(S+\overset{n}{\underset{i=1}{\sum }}\left(\frac{s_{i}}{k_{i}}\right)\right)+\overset{n}{\underset{i=1}{\sum }}h_{i}\left[\frac{1}{2}D_{i}\left(k_{i}T\right)+{\text{z}}_{i}\sqrt{\delta_{\text{i}}\left(k_{i}T+L_{i}\right)}\right]+\overset{n}{\underset{i=1}{\sum }}\frac{\pi_{i}}{k_{i}T}\sqrt{\delta_{\text{i}}\left(k_{i}T+L_{i}\right)}\left(f\left({\text{z}}_{i}\right)-{\text{z}}_{i}\left(1-F\left({\text{z}}_{i}\right)\right)\right). \end{array}$$

By derivation of TC with respect to z_*i*_, the following formula can be obtained:

(7) $$\begin{array}{c} \frac{\partial TC\left(K,T,z_{i}\right)}{\partial z_{i}}=h_{i}\sqrt{\delta_{i}\left(k_{i}T+L_{i}\right)}+\frac{\pi_{i}}{k_{i}T}\sqrt{\delta_{i}\left(k_{i}T+L_{i}\right)}\left(\frac{df\left({\text{z}}_{i}\right)}{d{\text{z}}_{i}}-\left[1-F\left({\text{z}}_{i}\right)\right]+{\text{z}}_{i}f\left({\text{z}}_{i}\right)\right). \end{array}$$

The standard normal distribution function satisfies *df*(z_*i*_)/*d*z_*i*_ = −z_*i*_*f*(z_*i*_). Therefore, we can get

(8) $$\begin{array}{c} \frac{\partial TC\left(K,T,z_{i}\right)}{\partial z_{i}}=\sqrt{\delta_{\text{i}}\left(k_{i}T+L_{i}\right)}\left(h_{i}-\frac{\pi_{i}}{k_{i}T}\left[1-F\left({\text{z}}_{i}\right)\right]\right). \end{array}$$

At the same time, if *∂TC*(*K*, *T*, *z*_*i*_)/*∂z*_*i*_ = 0, the optimal *z*_*i*_^∗^ must satisfy the following relation:

(9) $$\begin{array}{c} F\left({\text{z}}_{i}^{*}\left(K,T\right)\right)=1-\frac{h_{i}}{\pi_{i}}k_{i}T. \end{array}$$

Alternatively, it is written as an expression in the following inverse function form:

(10) $$\begin{array}{c} {\text{z}}_{i}^{*}\left(K,T\right)=F^{-1}\left(1-\frac{h_{i}}{\pi_{i}}k_{i}T\right). \end{array}$$

Because of $\partial^{2}TC\left(K,T,z_{i}\right)/\partial z_{i}^{2}=\left(\pi_{i}/k_{i}T\right)\sqrt{\delta_{i}\left(k_{i}T+L\right)}f\left(z_{i}\right)>0$, once *K* and *T* are determined, z_*i*_^∗^ can be uniquely obtained by formula (10). By substituting formula (10) into formula (7), we obtain the expression of the objective function TC(*K*, *T*, *z*_*i*_) of the stochastic JRP, as shown in

(11) $$\begin{array}{c} \min\text{TC}\left(K,T,z_{i}\right)=\overset{n}{\underset{i=1}{\sum }}\frac{1}{2}D_{i}h_{i}k_{i}T+\frac{1}{T}\left(S+\overset{n}{\underset{i=1}{\sum }}\left(\frac{s_{i}}{k_{i}}\right)\right)+\overset{n}{\underset{i=1}{\sum }}\frac{\pi_{i}}{k_{i}T}\sqrt{\delta_{i}\left(k_{i}T+L\right)}f\left(z_{i}\right). \end{array}$$

We build a JRP model based on RFID investment stochastic demand. First, we need to clarify the relationship between RFID technology investment cost and return. Due to the random uncertainty of demand, the capability of RFID technology is mainly reflected in the ability to improve the efficiency of joint procurement and reduce the cost of joint procurement. In order to distinguish the demand uncertainty JRP and the stochastic JRP after RFID investment in this section, we call the demand stochastic JRP as JRP1. Its corresponding total cost is TC1, and the random JRP of RFID investment demand is JRP2, and its corresponding total cost is TC2. The JRP decision model determined in this paper based on RFID technology is based on the JRP1 model. At the same time, referring to the RFID technology investment efficiency model, the JRP model of RFID investment is established. The model considers the impact of RFID on two costs of JRP, namely, the impact of ordering efficiency, and introduces the impact of efficiency factor R and inventory efficiency, which affects inventory cost and out-of-stock cost, and introduces JIT efficiency factor I.

The article "Application of Mathematical Modeling in Cost Control of Medical Equipment Procurement in Public Hospitals" was retracted in 2023. Reasons: unreliable results or conclusions; concerns about the data; concerns about the results or conclusions; concerns about the peer review.

After the ordering efficiency factor and the JIT efficiency factor are given, according to the equation, we get the total cost TC2 of the JRP model based on RFID technology to determine the demand:

(12) $$\begin{array}{c} \text{TC}2\left(T,K,z_{i},I,R\right)=I\cdot C_{H}+R\cdot C_{O}+I\cdot C_{S}+C_{I}+C_{R}=I\cdot \frac{T}{2}\overset{n}{\underset{i=1}{\sum }}k_{i}D_{i}h_{i}+R\cdot \frac{1}{T}\left(S+\overset{n}{\underset{i=1}{\sum }}\left(\frac{s_{i}}{k_{i}}\right)\right)+I\cdot \overset{n}{\underset{i=1}{\sum }}\frac{\pi_{i}}{k_{i}T}\sqrt{\delta_{i}\left(k_{i}T+L\right)}f\left(z_{i}\right)+C_{I}+C_{R}. \end{array}$$

It can be seen from the equation that if *I* = 1, it means that there is no JIT efficiency improvement for the JRP process. If *I* = 0, it means that the commodity order is completed immediately, no inventory cost occurs, and no out-of-stock cost occurs, and the “Justin Time” for customer service is realized. Similarly, if *R* = 1, it means that there is no improvement in ordering efficiency for JRP process by RFID technology. When *R* = 0, it means that the supply capacity is infinite, and no order cost occurs. In order to find the best relationship between *I* and *R*, the relationship between *I* and *C*_*I*_, and the relationship between *R* and *C*_*R*_, we need to build a functional expression that relates these relationships. The order efficiency function and the JIT efficiency function are, respectively, expressed as

(13) $$\begin{array}{c} I=V+\left(U-V\right)e^{-\lambda C_{l}}, \end{array}$$

(14) $$\begin{array}{c} R=N+\left(M-N\right)e^{-\beta C_{R}}. \end{array}$$

Among them, 0 ≤ *V* ≤ *U* ≤ 1, *U* is the lowest JIT efficiency, that is, the efficiency without RFID investment, and *V* is the highest efficiency after the implementation of RFID technology. 0 ≤ *N* ≤ *M* ≤ 1, *M* is the lowest efficiency of ordering, that is, the efficiency without RFID investment, and *N* is the highest efficiency after the implementation of RFID technology. Here, the determination of *U*, *V*, *M*, and *N* values can refer to the experience of RFID project implementation and can be estimated by investigating the impact of the use of RFID technology in related industries on efficiency. Among them, *λ*, *β* is the RFID investment efficiency control coefficient, which is used to adjust the RFID technology investment effect according to the actual RFID implementation.

The article "Application of Mathematical Modeling in Cost Control of Medical Equipment Procurement in Public Hospitals" was retracted in 2023. Reasons: unreliable results or conclusions; concerns about the data; concerns about the results or conclusions; concerns about the peer review.

In order to analyze the efficiency improvement produced by the investment in RFID technology, we bring equations (13) and (14) into equation (11); if TC2(*T*, *K*, *z*_*i*_, *I*, *R*) is differentiated with respect to *I* and set to zero, we can obtain the following equation:

(15) $$\begin{array}{c} \frac{\partial \text{TC}2\left(T,K,z_{i},I,R\right)}{\partial I}=C_{H}+C_{S}+\frac{\partial C_{I}}{\partial I}=C_{H}+C_{S}+\frac{1}{\lambda }\frac{\partial \left[\ln\left(U-V\right)-\ln\left(I-V\right)\right]}{\partial I}=C_{H}+C_{S}-\frac{1}{\lambda }\frac{1}{I-V}=0. \end{array}$$

From equation (15), if we can determine *C*_*H*_ and *C*_*S*_, we can get the optimal *I*^∗^:

(16) $$\begin{array}{c} I^{*}=\frac{1}{\lambda \cdot \left(C_{H}+C_{S}\right)}+V. \end{array}$$

Similarly, for equation (12), TC2(*T*, *K*, *z*_*i*_, *I*, *R*) takes the derivative of R and makes it zero, and if *C*_*O*_ can be determined, we can also obtain the optimal *R*^∗^:

(17) $$\begin{array}{c} R^{*}=\frac{1}{\beta \cdot C_{o}}+N. \end{array}$$

By constructing the JRP model (JRD1) under the condition of random demand and the JRP model of random demand based on RFID technology, the optimal *T*, *K*, *z*_*i*_, *I*, *R* is deduced. Next, we construct the DE solving algorithm based on the two stochastic demand JRP model structures, the number and type of decision variables.

The population length of the designed DE algorithm can be calculated in two ways. In the first way, all the decision variables can be randomly generated by the DE algorithm, but the range of each variable, especially *z*_*i*_, needs to be determined. The population length of the DE algorithm is the length of the combined procurement cycle of commodities, the length of the basic procurement cycle, and the length of the safety stock factor. The decision variables of the second method are derived from formulas, which are calculated with reference to formula (10) given the joint procurement period *K* and the basic procurement period *T* of different commodities.

The article "Application of Mathematical Modeling in Cost Control of Medical Equipment Procurement in Public Hospitals" was retracted in 2023. Reasons: unreliable results or conclusions; concerns about the data; concerns about the results or conclusions; concerns about the peer review.

The base purchase period is a decimal value between 0 and 1. The safety stock factor needs to consider the properties of the population of the normal distribution function, when the confidence level is 0.6827, *z*_*i*_ = 1.0, and when the customer service level is 99.99%, *z*_*i*_ ≈ 3.08. The level of customer service is determined according to the ability of the enterprise itself. Therefore, we can set the value range of 1 to 3, such as [1,3] or [1,2]. Under the second strategy, the search method of *K* and *T* can be completely referred to the content of Chapter 3, and then, the optimal combination of *K* and *T* is found and then the optimal *z*_*i*_ is calculated. For the sake of distinction, we call the JRP solution for the first strategy as JRP0 and the JRP solution for the second strategy as JRP1. Below, we set up the design process of the DE algorithm.

The solution process of the redesigned DE algorithm is also divided into the following three steps:

1. Parameter setting and initialization process

The algorithm parameters are divided into two categories: problem-related parameters and DE algorithm-related parameters. The problem parameter setting can refer to relevant research examples, and the DE algorithm parameter setting is based on the actual solution experience. The specific setting process is as follows:

- Problem parameter setting: we set the lower bound *k*_Lower_ and the upper bound *k*_Upper_ for each *k*_*i*_, respectively, and we set *k*_Lower_ = 1 and *k*_Upper_ = 5, where *i* = 1, 2, ⋯, *n*. At the same time, we design the initial value of *T* to be located at [0, 1], and the value range of *z*_*i*_ to be (1, 2).
- DE algorithm parameter setting: we set the DE algorithm population size pop, chromosome length l, mutation operator $\tilde{F}$, and crossover probability CR, respectively, and set t as the t-th generation population, and the objective function (total cost) as the fitness function fit. Since there are two initialization methods, the pp-th chromosome *e*_pp_ of the t-th generation population is initialized:

(18a) $$\begin{array}{c} {\text{chromosome}}_{\text{pp}}^{t}=\left(k_{1},k_{2},\cdots ,k_{n},T,z_{1},z_{2},\cdots ,z_{n}\right) \end{array}$$

Alternatively, the pp-th chromosome _pp_ of the t-th generation population is initialized as

(18b) $$\begin{array}{c} \text{ chromosom}{\text{e}}_{\text{pp}}^{t}=\left(k_{1},k_{2},\cdots ,k_{n},T\right). \end{array}$$

Among them, pp = 1, 2, ⋯, pop, the chromosome length under two different strategies is l = *n* + 1 or l = *n* + 1 + *n*. After these parameters are set, the algorithm goes to the next step to initialize the population.

(2) Initialize the population to calculate fitness and objective function values

Similar to the population initialization process of the DE algorithm in Chapter 3, if we define the algorithm population as *P*, the population is initialized as $P_{\text{pop}}^{t}=\left\{\left.X_{i}^{t}\right|x_{i,j}^{\text{lower}}\leq x_{i,j}^{t}\leq x_{i,j}^{\text{upper}},\tilde{i}=1,2,\cdots ,\text{pop};\tilde{j}=1,2,\cdots ,l;x_{\tilde{i},j}\left(t\right)\in X_{i}^{t}\right\}$. Among them, *x*_*i*,*j*_^lower^ = *K*^lower^/*T*^lower,^*x*_*i*,*j*_^upper^ = *K*^upper^/*T*^upper^, and when $\tilde{j}\leq n$, *x*_*i*,*j*_^*t*^ is usually calculated by

(19) $$\begin{array}{c} x_{\tilde{i},j}^{t=0}=\text{round}\left(x_{\tilde{i},j}^{\text{lower}}+\mathrm{rand}\left(0,1\right)\times \left(x_{\tilde{i},j}^{\text{upper}}-x_{\tilde{i},j}^{\text{lower}}\right)\right). \end{array}$$

Among them, “round” means rounding, and rand(0,1) is used to generate random numbers between (0,1).

The article "Application of Mathematical Modeling in Cost Control of Medical Equipment Procurement in Public Hospitals" was retracted in 2023. Reasons: unreliable results or conclusions; concerns about the data; concerns about the results or conclusions; concerns about the peer review.

Here, we still take the objective function as the fitness function. The calculation process of TC and TC1 refers to formula (11), and the calculation process of TC2 refers to formula (12). The purpose of population initialization is to generate the current optimal solution, the best fitness, and the chromosomes under the best fitness. These parameters are used in the update process of the DE algorithm.

(3) The main program of the DE algorithm runs

In order to better explain the flow of the DE algorithm, we take a four-commodity problem as an example to illustrate the three operations of the DE algorithm.

- Mutation operation: here, the t-th generation chromosome of the DE algorithm population is selected as the target vector of mutation. Within the range of the t-th generation population, three different integer numbers *r*_1_, *r*_2_, *r*_3_ that are different from the target vector are randomly generated, representing the *r*_1_-th, *r*_2_-th, and *r*_3_-th chromosomes of the population, respectively. If *I* presume mutation operator *F* = 0.4, then the whole mutation process according to the first strategy is shown in Figure 2. Figure 2 shows the schematic diagram of genes with multiple abnormal chromosomes after DE algorithm processing mutation. The basic processing idea is that if the mutated gene is abnormal, such as beyond the defined range, it will be replaced by a randomly generated qualified number. If the generated gene falls within the defined domain, the algorithm rounds the locus of $\tilde{j}\leq n$. Similarly, for the gene processing at $\tilde{j}>n$, if it exceeds the defined range, it is replaced by a randomly generated qualified number; otherwise, the calculated value of the variation formula is taken

(ii) Crossover operation: for each dimension, a vector with a length of 9 is randomly generated, which corresponds to the initial chromosome length of 9 (4 + 1 + 4), and a new chromosome is constructed with reference to expression (4-18a). If randn(*t*) = 4, CR = 0.4, new chromosomes will be generated according to the quantum crossover rule, as shown in Figure 3

(iii) Algorithm selection and update operations: according to the greedy selection rule, the selection operation of the DE algorithm is performed, the fitness of each chromosome is calculated, and the current optimal fitness and the current optimal chromosome are output
(iv) The algorithm repeats algorithm steps (1)-(3) until the maximum number of iterations is reached or the algorithm converges
(v) The algorithm outputs the optimal result
(vi) When the maximum number of iterations is reached, the DE algorithm stops running and outputs the best fitness, the chromosome corresponding to the best fitness, and the optimal solution

The flow chart of DE algorithm to solve the random demand JRP is shown in Figure 4.

The article "Application of Mathematical Modeling in Cost Control of Medical Equipment Procurement in Public Hospitals" was retracted in 2023. Reasons: unreliable results or conclusions; concerns about the data; concerns about the results or conclusions; concerns about the peer review.

## 4. Cost Control System for Medical Equipment Procurement in Public Hospitals

Through the business demand analysis and data analysis of the medical equipment quota management system in the opposite hospital, various business flow charts have been used to clearly show the current equipment supply management business process. Therefore, the function that the system should achieve can be derived. Its functional modules include user login module, planning module, auditing module, equipment ordering module, storage and outgoing module, payment module, statistical query module, and equipment supplier data module. The specific functions that can be realized are as follows: (1) user login: it is used to verify the user's identity and access rights to determine their operation rights. (2) Plan input: it is used for the input of equipment plan. (3) Audit module: it is used to verify whether the equipment plan is reasonable. (4) Equipment order: it is used by the business department to input various information related to equipment into the system. (5) Inbound and outbound: it is used for the management of equipment arrival, inbound, outbound, etc. by business departments and equipment users. (6) Payment: it supports input, statistics, and inquiry of expenses for equipment. (7) Statistical query: it is used for different needs of different users and can flexibly check and count data information related to the equipment. (8) Equipment supplier data: it is used for the access, approval, and annual evaluation of suppliers. The connection between modules is shown in Figure 5.

The article "Application of Mathematical Modeling in Cost Control of Medical Equipment Procurement in Public Hospitals" was retracted in 2023. Reasons: unreliable results or conclusions; concerns about the data; concerns about the results or conclusions; concerns about the peer review.

As can be seen from Figure 6, the equipment management and procurement management platforms of public hospitals can be roughly divided into supplier management, equipment management and procurement management, and waste equipment management according to the order of equipment circulation.

After further refining the three-layer structure, the public hospital equipment management and procurement management information platform can be divided into five subsystems: equipment management system, supplier management system, procurement management system, spare parts management system, and waste equipment management system. The platform not only realizes the equipment safety management but also realizes the informatization of equipment procurement, so that the coal enterprises can greatly improve the continuous production capacity of the enterprises while producing safely. At the same time, purchasing equipment or accessories through online bidding not only ensures the quality of equipment or accessories but also greatly saves the procurement cost of enterprises. The architecture diagram of the equipment management and procurement management information platform is shown in Figure 7.

The conceptual model of the system is the theoretical basis of the equipment procurement cost control system and the most fundamental theoretical basis for the construction of the system. This construction is based on the optimization of the conceptual model of strategic procurement, changes the cooperation mode of the project, and replaces the bargaining based on the traditional procurement management theory by strategic cooperation. On the other hand, based on the theoretical model of value creation based on lean construction, the control method of the project is transformed, and the task management based on the transformation theoretical model is replaced by value management. The overall framework of the equipment procurement cost control system is shown in Figure 8.

On this basis, the effect of the model proposed in this paper is verified, and the procurement cost control effect of the model in this paper is counted. The results are shown in Table 1 and Figure 9.

From the analysis of the above chart data, we can see that the cost control system for medical equipment procurement in public hospitals based on mathematical modeling proposed in this paper can play an important role in equipment procurement in public hospitals.

## 5. Conclusion

Under the development situation of the new medical reform, my country has made major reforms in improving the procurement quality and efficiency standards of public hospitals, which has achieved the steady development of hospital business and promoted the transformation of hospitals from extensive management to refined management. In the management of large-scale medical equipment, by evaluating the benefits of large-scale medical equipment, the use efficiency of the equipment can be clarified, and it can also provide reference for the planning and project establishment of large-scale medical equipment. The benefit evaluation of the hospital's medical equipment before the purchase can judge the benefit of the capital investment, evaluate whether the investment is feasible, and prevent the waste of funds and idle equipment. Combined with the procurement process of medical equipment in public hospitals, this paper establishes a mathematical model of medical equipment procurement in public hospitals. Data analysis shows that the cost control system for medical equipment procurement in public hospitals based on the mathematical model proposed in this paper can play an important role in public hospital equipment procurement.

The article "Application of Mathematical Modeling in Cost Control of Medical Equipment Procurement in Public Hospitals" was retracted in 2023. Reasons: unreliable results or conclusions; concerns about the data; concerns about the results or conclusions; concerns about the peer review.

## Figures and Tables

**Figure 1:** Schematic diagram of the JRP model under random demand conditions.

**Figure 2:** Schematic diagram of mutation operation.

**Figure 3:** Schematic diagram of crossover operation.

**Figure 4:** Flowchart of the DE algorithm.

**Figure 5:** Equipment supply management system.

**Figure 6:** Schematic diagram of the procurement management information platform process.

**Figure 7:** Architecture diagram of procurement management information platform.

**Figure 8:** Overall framework of equipment procurement cost control system.

**Figure 9:** Statistical diagram of the effect of the cost control system for medical equipment procurement in public hospitals based on mathematical modeling.

**Table 1:** Statistical table of the effect of the cost control system for medical equipment procurement in public hospitals based on mathematical modeling.

No.	Cost control	No.	Cost control	No.	Cost control
1	81.421	20	83.748	39	88.994
2	83.906	21	79.917	40	88.236
3	85.060	22	85.896	41	91.460
4	86.548	23	80.946	42	82.206
5	89.309	24	89.212	43	86.927
6	91.146	25	82.835	44	90.777
7	87.050	26	90.513	45	82.321
8	84.836	27	91.314	46	83.567
9	82.388	28	81.307	47	82.499
10	80.449	29	91.543	48	80.325
11	82.452	30	79.152	49	91.302
12	90.958	31	84.065	50	86.035
13	89.631	32	89.820	51	87.832
14	83.687	33	85.314	52	81.333
15	85.705	34	80.048	53	88.433
16	89.994	35	89.002	54	88.910
17	82.295	36	87.456	55	83.767
18	80.719	37	85.653	56	80.221
19	85.524	38	82.464		

## Data Availability

The labeled dataset used to support the findings of this study are available from the corresponding author upon request.
